# The Rise of Cloud Computing: Data Protection, Privacy, and Open Research Challenges—A Systematic Literature Review (SLR)

**DOI:** 10.1155/2022/8303504

**Published:** 2022-06-07

**Authors:** Junaid Hassan, Danish Shehzad, Usman Habib, Muhammad Umar Aftab, Muhammad Ahmad, Ramil Kuleev, Manuel Mazzara

**Affiliations:** ^1^Department of Computer Science, National University of Computer and Emerging Sciences, Islamabad, Chiniot-Faisalabad Campus, Chiniot 35400, Pakistan; ^2^Department of Computer Science, Superior University, Lahore 54000, Pakistan; ^3^Faculty of Computer Sciences and Engineering, GIK Institute of Engineering Sciences and Technology, Topi, Swabi 23640, Khyber Pakhtunkhwa, Pakistan; ^4^Institute of Software Development and Engineering, Innopolis University, Innopolis 420500, Russia

## Abstract

Cloud computing is a long-standing dream of computing as a utility, where users can store their data remotely in the cloud to enjoy on-demand services and high-quality applications from a shared pool of configurable computing resources. Thus, the privacy and security of data are of utmost importance to all of its users regardless of the nature of the data being stored. In cloud computing environments, it is especially critical because data is stored in various locations, even around the world, and users do not have any physical access to their sensitive data. Therefore, we need certain data protection techniques to protect the sensitive data that is outsourced over the cloud. In this paper, we conduct a systematic literature review (SLR) to illustrate all the data protection techniques that protect sensitive data outsourced over cloud storage. Therefore, the main objective of this research is to synthesize, classify, and identify important studies in the field of study. Accordingly, an evidence-based approach is used in this study. Preliminary results are based on answers to four research questions. Out of 493 research articles, 52 studies were selected. 52 papers use different data protection techniques, which can be divided into two main categories, namely noncryptographic techniques and cryptographic techniques. Noncryptographic techniques consist of data splitting, data anonymization, and steganographic techniques, whereas cryptographic techniques consist of encryption, searchable encryption, homomorphic encryption, and signcryption. In this work, we compare all of these techniques in terms of data protection accuracy, overhead, and operations on masked data. Finally, we discuss the future research challenges facing the implementation of these techniques.

## 1. Introduction

Recent advances have given rise to the popularity and success of cloud computing. It is a new computing and business model that provides on-demand storage and computing resources. The main objective of cloud computing is to gain financial benefits as cloud computing offers an effective way to reduce operational and capital costs. Cloud storage is a basic service of cloud computing architecture that allows users to store and share data over the internet. Some of the advantages of cloud storage are offsite backup, efficient and secure file access, unlimited data storage space, and low cost of use. Generally, cloud storage is divided into five categories: (1) private cloud storage, (2) personal cloud storage, (3) public cloud storage, (4) community cloud storage, and (5) hybrid cloud storage.

However, when we outsource data and business applications to a third party, security and privacy issues become a major concern [1]. Before outsourcing private data to the cloud, there is a need to protect private data by applying different data protection techniques, which we will discuss later in this SLR. After outsourcing the private data to the cloud, sometimes the user wants to perform certain operations on their data, such as secure search. Therefore, while performing such operations on private data, the data needs to be protected from intruders so that intruders cannot hack or steal their sensitive information.

Cloud computing has many advantages because of many other technical resources. For example, it has made it possible to store large amounts of data, perform computation on data, and many other various services. In addition, the cloud computing platform reduces the cost of services and also solves the problem of limited resources by sharing important resources among different users. Performance and resource reliability requires that the platform should be able to tackle the security threats [2]. In recent years, cloud computing has become one of the most important topics in security research. These pieces of research include software security, network security, and data storage security.

The National Institute of Standards and Technology (NIST) defines cloud computing as [3] “a model for easy access, ubiquitous, resource integration, and on-demand access that can be easily delivered through various types of service providers. The Pay as You Go (PAYG) mechanism is followed by cloud computing, in which users pay only for the services they use. The PAYG model gives users the ability to develop platforms, storage, and customize the software according to the needs of the end-user or client. These advantages are the reason that the research community has put so much effort into this modern concept [4].

Security is gained by achieving confidentiality, integrity, and data availability. Cloud users want assurance that their data must be saved while using cloud services. There are various types of attacks that launch on a user's private data, such as intrusion attacks, hacking, stealing the user's private data, and denial of service attacks. 57% of companies report security breaches using cloud services [5]. Data privacy is more important than data security because cloud service providers (CSPs) have full access to all cloud user's data and can monitor their activities, because of which the cloud user privacy is compromised. For example, a user is a diabetic, and the CSP is analyzing their activities, such as what he is searching for more and what kind of medicine he is using the most. Because of this access, CSP can get all the sensitive information about an individual user and can also share this information with a medicine company or an insurance company [6]. Another problem is that the user cannot fully trust CSP. Because of this reason, there are many legal issues. Users cannot store their sensitive data on unreliable cloud services because of this mistrust. As a result, many users cannot use cloud services to store their personal or sensitive data in the cloud. There are two ways to solve this problem. One is that the user installs a proxy on his side, and this proxy takes the user's data, encrypts and saves their data using some data protection techniques, and then sends it to the untrusted CSP [7].

The recent Google privacy policy is that any user can use any Google service free of cost; however, Google monitors their activity by monitoring their data to improve their services [8]. In this paper, we compare different types of data protection techniques that provide privacy and security over the data stored on the cloud. Many papers discuss outsourcing data storage on the cloud [9, 10], however, we also discuss how we can secure the outsourced data on the cloud. Most of the paper describes the data security on the cloud vs the external intruder attacks [11, 12]. This paper not only discusses the security attacks from outside intruders and securing mechanisms but also inner attacks from the CSP itself. Many surveys cover data privacy by applying cryptographic techniques [13, 14]. These cryptographic techniques are very powerful for the protection of data and also provide a very significant result. However, there is a problem as these cryptographic techniques require key management, and some of the cloud functionalities are not working on these cryptographic techniques. In this paper, we also discuss some steganographic techniques. To the best of our knowledge, no study discusses all the conventional and nonconventional security techniques. Therefore, all the data protection techniques need to be combined in one paper.

The rest of this paper is organized as follows: Section 3 of the paper describes the research methodology that consists of inclusion, exclusion criteria, quality assessment criteria, study selection process, research questions, and data extraction process. Also, we discuss assumptions and requirements for data protection in the cloud.  Section 4 presents all the cryptographic and also noncryptographic techniques that are used for data protection over the cloud. Also, we discuss the demographic characteristics of the relevant studies by considering the following four aspects: (i) publication trend, (ii) publication venues (proceeding and journals), (iii) number of citations, and (iv) author information.  Section 4 also compares all these data protection techniques. Lastly, in Section 5, we discuss results and present conclusion and future work.

## 2. Related Work

The first access control mechanism and data integrity in the provable data possession (PDP) model is proposed in the paper [15], and it provides two mobile applications based on the RSA algorithm. Like the PDP, the author in the paper [16] proposed a proof of retrievability (PoR) scheme that is used to ensure the integrity of remote data. PoR scheme efficiency is improved using a shorter authentication tag that is integrated with the PoR system [17]. A more flexible PDP scheme is proposed by the author of the paper [18] that uses symmetric key encryption techniques to support dynamic operations. A PDP protocol with some flexible functionality is developed, in which, we can add some blocks at run time [19]. A new PDP system with a different data structure is introduced, and it improves flexibility performance [20]. Similarly, another PDP model with a different data structure is designed to handle its data functionality [21]. To improve the accuracy of the data, the author of the paper [22] designed a multireplicas data verification scheme that fully supports dynamic data updates.

A unique data integration protocol [23] for multicloud servers is developed. The author of the paper [24] also considers the complex area where multiple copies are stored in multiple CSPs and builds a solid system to ensure the integrity of all copies at once. A proxy PDP scheme [25] is proposed, which supports the delegation of data checking that uses concessions to verify auditor consent. In addition, the restrictions of the verifier are removed that strengthened the scheme, and it proposes a separate PDP certification system [26]. To maintain the security of information, a concept for information security is proposed and a PDP protocol for public research is developed [27]. To resolve the certification management issue, the PDP system with data protection is introduced [28].

Identity-based cryptography is developed, in which a user's unique identity is used as input to generate a secret key [29]. Another PDP protocol is recommended to ensure confidentiality [30]. The author of the paper [31] proposed a scheme, in which tags are generated through the ring signature technique for group-based data sharing that supports public auditing and maintains user privacy. A new PDP system is introduced for data sharing over the cloud while maintaining user privacy [32]. Additionally, it supports the dynamic group system and allows users to exit or join the group at any time. Another PDP system [33] that is based on broadcast encryption and supports dynamic groups [34] is introduced. The issue of user revocation has been raised [35], and to address this issue, a PDP scheme has been proposed, which removes the user from the CSP using the proxy signature method. A PDP-based group data protocol was developed to track user privacy and identity [36]. A PDP system [37] is proposed for data sharing between multiple senders. The author of the paper [38] provides SEPDP systems while maintaining data protection. However, the author of the paper [39] proved that the scheme proposed in [38] is vulnerable to malicious counterfeiting by the CSP. A collision-resistant user revocable public auditing (CRUPA) system [40] is introduced for managing the data that is shared in groups. Another scheme [41] is introduced as a way to ensure the integrity of mobile data terminals in cloud computing.

To address the PKI issue, identity-based encryption [42] is designed to enhance the PDP protocol and maintain user privacy in a dynamic community. Before sharing user-sensitive data with third parties or researchers, data owners ensure that the privacy of user-sensitive data is protected. We can do this using data anonymization techniques [43]. In recent years, the research community has focused on the PPDP search area and developed several approaches for tabular data and SN [44–49]. There are two popular settings in PPDP: one is interactive, and the other is noninteractive [50]. The K-anonymity model [51] and its effects are most commonly used in the noninteractive setting of PPDP [52–56]. Differential privacy (DP) [57] and an interactive configuration of PPDP make extensive use of DP-based methods [58–60]. Meanwhile, several studies for a noninteractive setting reported a PD-dependent approach [61]. Researchers have expanded the concepts used to anonymize tabular data to protect the privacy of SN users [62–64].

Most images on the internet are in a compressed form. Hence, various studies design some techniques for AMBTC-compressed images. Data concealment has become an active research area. We can hide the data by adding confidential information to the cover image, and as a result, we get the stego image. There are two types of data hiding schemes: one is irreversible [65–68], and the other is a reversible data hiding scheme [69–71]. A cipher text designated for data collection can be re-encrypted as designated for another by a semitrusted proxy without decryption [72]. The first concrete construction of collusion-resistant unidirectional identity-based proxy re-encryption scheme, for both selective and adaptive identity, is proposed in the paper [73]. One of the data hiding schemes is the histogram shifting scheme [74–76], and it is the most widely used. A histogram-shifting data hiding scheme [77] that detects pixel histograms in the cover image is introduced. When big and diverse data are distributed everywhere, we cannot control the vicious attacks. Therefore, we need a cryptosystem to protect our data [78–80].

Some identity-based signature (IBS) schemes [81–84] are introduced that are based on bilinear pairing. However, the authentication schemes based on bilinear pairing over elliptic curve are more efficient and safer than traditional public key infrastructure [85, 86]. The paper [87] proposed a preserving proxy re-encryption scheme for public cloud access control. A differential attack is performed on one-to-many order preserving encryption OPE by exploiting the differences of the ordered ciphertexts in [88]. Another scheme is proposed, which consists of a cancelable biometric template protection scheme that is based on the format-preserving encryption and Bloom filters [89]. Some of the researchers also use the concept of paring free identity-based signature schemes [90–93]. A lightweight proxy re-encryption scheme with certificate-based and incremental cryptography for fog-enabled e-healthcare is proposed in [94].

## 3. Research Methodology

The objective of this SLR is to evaluate, investigate, and identify the existing research in the context of data storage security in cloud computing to find and evaluate all the existing techniques. SLR is a fair and unbiased way of evaluating all the existing techniques. This way provides a complete and evidence-based search related to a specific topic. At this time, there is no SLR conducted on data storage security techniques that explains all the cryptographic and noncryptographic techniques. Hence, this SLR fulfills the gap by conducting itself. This SLR aims to provide a systematic method using the guidelines of an SLR provided by Kitchenham [95]. Furthermore, to increase the intensity of our evidence, we follow another study that is provided by [96]. Our SLR consists of three phases, namely planning, conducting, and reporting. By following these three phases, we conduct our SLR, as shown in Figure 1.

### 3.1. Research Questions

The primary research question of this systematic literature review is “What types of data protection techniques have been proposed in cloud computing?” This primary research question is further divided into four RQs. All these four questions are enlisted below.

  RQ1: what types of data protection techniques have been proposed in cloud computing?
  RQ2: what are the demographic characteristics of the relevant studies?
  RQ3: which data protection technique provides more data protection among all the techniques?
  RQ4: what are the primary findings, research challenges, and directions for future research in the field of data privacy in cloud computing?

### 3.2. Electronic Databases

Six electronic databases were selected to collect primary search articles. All these six electronic databases are well-reputed in the domain of cloud computing. Most of the relevant articles are taken from two electronic databases, namely IEEE and Elsevier. All the electronic databases that we use in this research process are given in Table 1.

### 3.3. Research Terms

First of all, the title base search is done on the different electronic databases, which are given in Table 1. After that, most related studies/articles are taken. Search is done using the string (p1 OR p2. . . . . .OR pn.) AND (t1 OR t2. . . . . . OR tn.). This string/query is constructed using a population, intervention, control, and outcomes (PICO) structure that consists of population, intervention, and outcome. Database search queries are given in Table 2.

 
*Population*: “cloud computing”
 
*Intervention*: “data security,” “data privacy,” “data integrity”
  Using the PICO structure, we construct a general query for the electronic database. *Generic: ((“Document Title”: cloud∗) AND (“Document Title”: data AND (privacy OR protect∗ OR secure∗ OR integrity∗))).*

### 3.4. Procedure of Study Selection

The procedure of study selection is described in Figure 2. This procedure has three phases: the first one is exclusion based on the title, in which articles are excluded based on the title, and the relevant titles are included. The second is exclusion based on the abstract in which articles are excluded. By reading the abstract of the articles, the most relevant abstract is included, and the last one is exclusion based on a full text that also includes quality assessment criteria.

### 3.5. Eligibility Control

In this phase, all the selected papers are fully readied, and relevant papers are selected to process our SLR further.  Table 3 shows the final selected papers from each database based on inclusion and exclusion criteria. The related papers are selected based on inclusion and exclusion criteria, which are given in Table 4.

### 3.6. Inclusion and Exclusion Criteria

We can use the inclusion and exclusion criteria to define eligibility for basic study selection. We apply the inclusion and exclusion criteria to those studies that are selected after reading the abstract of the papers. The criteria for inclusion and exclusion are set out in Table 4. Table 4 outlines some of the conditions that we have applied to the articles. After applying the inclusion and exclusion criteria, we get relevant articles, which we finally added to our SLR. The search period is from 2010 to 2021, and most of the papers included in our SLR are from 2015 to onward.

We apply inclusion and exclusion criteria in the third phase of the study selection process, and we get 139 results. After that, we also apply quality criteria, and finally, we get 52 articles, which are included in this SLR. Most of the articles are taken from Elsevier and IEEE electronic databases. IEEE is the largest Venus for data storage security in cloud computing. The ratio of the selected articles from different electronic databases is shown in Figure 3.

### 3.7. Quality Assessment Criteria

Quality checking/assessment is done in the 3^rd^ phase of the study selection process. A scale of 0-1 is used for the quality assessment (QA) of the articles.

Poor-quality articles get 0 points on the scale, and good-quality articles get 1 point on the scale. The articles with 1 point on the scale are included in this SLR. Hence, by applying the quality checking/assessment criteria on all the articles, we finally get 52 articles. All the selected papers have validity and novelty for different data protection techniques, and also, we find the relevance of the articles in the quality assessment criteria, which ensures that all the articles are related to the SLR (data storage protection and privacy in cloud computing). The quality checking (QC) criteria are given in Table 5.

### 3.8. Taxonomy of the Data Protection Techniques

In this section, all the data protection techniques are depicted in Figure 4. All the data protection techniques are arranged and classified in their related categories. The purpose of the taxonomy is to give a presentational view of all the data protection techniques. The data protection techniques are mainly divided into two categories, namely (1) noncryptographic techniques and (2) cryptographic techniques.

## 4. Results and Discussions

Data protection on the cloud is done by developing a third-party proxy that is trusted by the user. The trusted proxy is not a physical entity. It is a logical entity that can be developed on the user end (like on the user's personal computer) or at that location on which the user can trust. Mostly, all the local proxies are used as an additional service or as an additional module (like browser plugins). To fulfill the objective of data protection by proxies, some requirements are needed to fulfill necessarily. The requirements are given below:

1. User privilege. There are several objectives of user privilege or user empowerment, however, the main objective is to increase the trust of the users in data protection proxies used by the cloud.
2. Transparency. Another important objective is that when users outsource their sensitive data to trusted proxies, their data should remain the same and should not be altered.
3. Cloud computing provides large computing power and cost saving resources. However, one concern is that if we increase data security, computation overhead should not increase. We want to minimize the computation overhead over the proxies.
4. Cloud functionalities preservation. Cloud functionalities preservation is the most important objective. The users encrypt their sensitive data on their personal computers by applying different encryption techniques to increase the protection of their data, however, by applying these different encryption techniques, they are not able to avail some of the cloud functionalities because of compatibility issues [97]. Hence, it is the main issue.

Figure 5 provides a data workflow for protecting sensitive data on the cloud using a local proxy. There are different types of the assumption that are made for data protection, and some of them are discussed below.

- Curious CSPs, the most commonly used model in cloud computing, is given in the literature [98]. The cloud service provider honestly fulfills the responsibilities, i.e., they do not interfere in the user activities, and they only follow the stander protocols. The CSP is honest, however, sometimes, it is curious to analyze the users' queries and analyze their sensitive data, which is not good because it is against the protocol. Also, by this, the privacy of the user is compromised. Hence, we can avoid these things by applying some data protection techniques on the user end to protect the users' sensitive data from the CSPs.
- In some cases, CSPs may collaborate with data protection proxies that are present on the users' sides to increase the level of trust between the users and CSPs because better trust can motivate more users to move to the cloud. This collaboration can be done if CSPs provide some services to the users with a stable interface for storing, searching, and computing their data.
- A multicloud approach to cloud computing infrastructure has also been proposed to improve their performance. In this regard, multiple cloud computing services are provided in the same heterogeneous architecture [19]. A multicloud gives the user multiple different places to store their data at their desired location. There are several benefits to use a multicloud, e.g., it reduces reliance on a single CSP, which increases flexibility.

### 4.1. RQ1: What Type of Data Protection Techniques has Been Proposed in Cloud Computing?

In this session, we will discuss all the techniques for data storage security over the cloud. All these techniques are divided into two main categories, namely (i) cryptographic techniques and (ii) noncryptographic techniques. The local proxy uses different techniques to protect data that are stored on the cloud. Because of this reason, we cannot gain all the advantages of cloud services. Therefore, we analyze and compare all these techniques based on different criteria. These different criteria are as follows: (i) the data accuracy of all the techniques, (ii) the data protection level of all the techniques, (iii) all the functionalities these schemes allow on masked and unmasked data, and (iv) the overhead to encrypt and decrypt data over the cloud.

#### 4.1.1. Noncryptographic Techniques

There are some noncryptographic techniques, and we discuss them in this paper as follows:

*(1) Data Anonymization*. Data anonymization is a data privacy technique used to protect a user's personal information. This technique hides the person's personal information by hiding the person's identifier or attributes that could reveal a person's identity. Data anonymization can be done by applying various mechanisms, for example, by removing or hiding identifiers or attributes. It can also be done by encrypting the user's personal information. The main purpose of performing data anonymization is that we can hide the identity of the person in any way. Data anonymity can be defined as the user's personal data being altered in such a way that we cannot directly or indirectly identify that person, and the CSP cannot retrieve any person's personal information. Data anonymization techniques have been developed in the field of statistical control disclosure. These techniques are most often used when we want to outsource sensitive data for testing purposes. Data anonymization is graphically represented in Figure 6.

Data anonymization techniques are most often used when we want to outsource sensitive data for testing purposes. For example, if some doctors want to diagnose certain diseases, some details of these diseases are required for this purpose. This information is obtained from the patients that suffer from these diseases, but it is illegal to share or disclose anyone's personal information. However, for this purpose, we use data anonymization technique to hide or conceal the person's personal information before outsourcing the data. In some cases, however, the CSP wants to analyze the user's masked data. In the data anonymization technique, attributes are the most important part. Attributes can include name, age, gender, address, salary, etc.  Table 6 shows the identifiers classification.

Data anonymization can be performed horizontally or vertically on this table and also on the record or group of records. The attributes are further classified into the following categories.

- Sensitive Attributes: sensitive attributes possess sensitive information of the person, such as salary, disease information, phone number, etc. These attributes are strongly protected by applying some protection techniques.
- Nonsensitive Attributes: these types of attributes do not belong to any type of category. Hence, they do not disclose the identity of a person.
- Identifiers: identifier belongs to the identity of a person, such as Id card, name, social security number, etc. Because of the presence of these identifiers, the relationship between different attributes can be detected. Hence, these identifiers must be replaced or anonymized.
- Quasi-Identifiers: quasi-identifiers are the group of identifiers that are available publicly, such as zip-code, designation, gender, etc. Separately, these identifiers cannot reveal the personal identity, however, by combining them, they may reveal the identity of the person. Hence, we want to separate these quasi-identifiers to avoid the discloser.

There are two main categories of data masking: (1) perturbative masking and (2) nonperturbative masking.

(1) *Perturbative Masking*
In perturbation, masking data is altered or masked with dummy datasets. Original data is replaced with dummy data, however, this data looks like the original data with some noise addition. The statistical properties of the original data are present in the masked data, however, nonperturbative masking does not contain the statistical properties of original data, because in perturbation masking, data is altered or masked with physically same but dummy data.
Some of the perturbative masking methods are given below.
  - *Data swapping*
  - In data swapping, the data is randomly changed with the same but dummy data between different records [99]. However, if the numerical values are present in the dataset, then in certain limits, the values can be changed. Otherwise, the meaning of the data is changed. The masked data cannot look like the original data. For those attributes that can be ranked, the attribute is replaced with the nearby ranked attributes, and a very large difference between ranks is not suitable [100]. In data swapping, higher-level attributes are swapped [101] and individual values are not changed.
  - *Noise Addition*
  - In this mechanism, some noise is added to the original dataset to alter the original data. Noise is only added to the data that is continuous and divided into categories [102]. The noise is added into all the attributes that are present in the original dataset, such as sensitive attributes and also quasi-attributes.
  - *Microaggregation*
  - In this technique, all the relevant data is stored into different groups, and these different groups release average values from each record [103]. If a large number of similar records is present in different groups, then more data utility is done. We can cluster the data in many ways, e.g., in categorical versions [104]. Microaggregation is done on a quasi-attribute to protect these attributes from reidentification, and the quasi-attributes protect all the other attributes from reidentification. We can also minimize reidentification by data clustering [105].
  - *Pseudonymization*
  - In this method, the original data is replaced with artificial datasets [106]. In this technique, each attribute present in the original data is a pseudonym, and by doing this, data is less identifiable.
(2) Nonperturbative Masking
Nonperturbative masking does not change or alter the original data, however, it changes the statistical properties of the original data. Mask data is created by the reduction of the original data or suppressions of the original data [107].
Some methods that are used for nonperturbative masking are as follows:
  - *Bucketization*
  - In this method, original data is stored in different buckets, and these buckets are protected through encryption [108]. We can protect the sensitive attributes through bucketization.
  - *Slicing*
  - Data slicing is a method in which a larger group of data is divided into smaller slices or segments [109]. Hence, we can slice the data, and in this way, the sensitive attribute and the quasi-attributes are divided into different slices. By identifying the individual slice, the identity of the person cannot be disclosed.
  - *Sampling*
  - Sampling is a technique in which the population and sample concept is present. The entire data is called population, and the masked data is called a sample. In this technique, we make different samples of the original data. A smaller data sample provides more protection [110].
  - *Generalization*
  - It is a technique in which some additional attributes are added to the record. If the number of quasi-attributes is less rare, then some dummy attributes are added into the record, which look like the quasi-attributes. Hence, by doing this, reidentification becomes more difficult [111]. By applying generalization on data, we can protect the identity of a person because it hides the relationship between the quasi-attributes.

The summary of data anonymization techniques is given in Table 7.

*(2) Data Splitting*. Data splitting is a technique in which sensitive data is divided into different fragments [112] to protect it from unauthorized access. In this technique, we first split the data into different fragments, then these fragments are randomly stored on different clouds. Even if the intruder gains access to a single fragment in any way, still the intruder will not be able to identify the person. For example, if an intruder gets a fragment from the cloud that contains the salary information of an organization, it is useless until he knows which salary belongs to which person. Hence, data splitting is a very useful technique for protecting data stored on the cloud.

Local proxies outsource data to the cloud without splitting the data, and they can also split the data first and then outsource to the same cloud using different accounts in the same CSP. It can also store data on different cloud platforms that run through different CSPs but provide some of the same services. Data is split before storing in different locations because even if some part or piece of data is known to an intruder, they will not be able to identify anyone.

Firstly, the local proxy retrieves sensitive data from the user and then calculates the risk factor for disclosure. In this method, the user can define the privacy level, and this privacy level provides information about all the sensitive attributes that can reveal someone's identity. These sensitive attributes are called quasi-attributes or quasi-identifiers. Next, the local proxy decides the number of pieces into which the sensitive data will be split and the number of locations that will be needed to store those pieces. Therefore, no one can reveal a person's identity, and all this information about the data splitting mechanism is stored at the local proxy. However, the system must be able to function properly and respond to the queries on time. After that, the local proxy stores these different data fragments in different cloud databases, and now, they are free from disclosure. The data-splitting mechanism supports almost all the functions of the cloud. Hence, we can use almost all the services provided by CSP using the data-splitting mechanism for storing data in the cloud.

When the users want to retrieve the original data, they process a query on a local proxy. The query is processed, and the data storage locations are retrieved from the local database. After that, the query is replicated as many times as the data is split into fragments, and these queries are forwarded to the relevant CSPs. As a result, each CSP provides a set of results that represent a partial view of the complete result. Finally, the proxy collects partial results according to the criteria used to split the data and provides the complete result to the user. Mostly, all these fragments are stored on different cloud databases in their original structure. Therefore, computation on these fragments can be performed easily. However, there is a problem if we want to perform computation separately on the individual fragment. Then, there is no algorithm that exists for this computation. Therefore, some algorithms are required to perform these types of computation as this computation requires communication between different CSPs. The redundancy of proxy metadata and backup policies must be essential to ensure the robustness of the mechanism. The data-splitting is graphically represented in Figure 7.

The summary of the data-splitting is given in Table 8. Different data-splitting techniques are used for the protection of data stored on the cloud. Some of these are given below.

- *Byte level splitting*
- In this type, all the sensitive data is converted into bytes [113]. Then, these bytes are randomly shuffled with each other. After that, all the bytes are recombined. Fixed length fragments are made, and then, these fragments are stored on a different cloud.
- *Privacy level splitting*
- In this mechanism, the user chose the privacy level of each file [114] that is to be stored on a cloud database. Hence, a privacy level is attached with the file that is to be stored on the cloud. Using this privacy level, the user can decide that the higher privacy level files should be stored on the trusted cloud.
- *Byte level splitting with replication*
- Byte-level data splitting is combined with data replication to improve both performance and security. The author of the paper [115] proposed an algorithm to store the data fragments on different clouds, so that they are at a certain distance and by doing this; we can avoid confabulation attacks where the intruder can aggregate the split fragments.
- *Byte level splitting with encryption*
- Firstly, byte-level data splitting [116, 117] is proposed. In this scheme, every fragment of data is encrypted to enhance the security of sensitive data. In this mechanism, the data is split into bytes, and these bytes are randomly shuffled and finally recombined. This type of data splitting is suitable for binary or multimedia files that are not processed through the cloud.
- Another problem is the length of a fragment in which we can say that the data cannot be reidentified or the identity of a person cannot be revealed. If the length is too short, then the probability of disclosure increases, and if the length is too long, then it is difficult to handle these fragments. Hence, it should have a certain length so that we can also protect the identity of a person.
- There is another type of data splitting in which we split data into attributes. The attribute level splitting is performed in two ways: one is horizontal splitting and the second is vertical splitting. These types of splitting are mostly done on structural databases, and they provide strong privacy.
- *Vertical splitting*
- In vertical data splitting [118, 119], we divide quasi-identifiers or quasi-attributes in such a way that all the risky attributes are divided into different fragments to secure the reidentification. Some of the sensitive fragments required encryption on it. Hence, we can encrypt these fragments by applying some encryption algorithms or by applying some other privacy methods to increase the security level.

A solution for sensitive data splitting without performing encryption on fragments is proposed [120]. This mechanism is suitable for data on which we want to perform some computation, because on encrypted data, we cannot perform computation directly. Another technique has been proposed [121], which demonstrates the redaction and sanitization of a document that identifies all sensitive attributes and protects the data in most documents.

The schemes that use vertical splitting to protect data are faster than other splitting techniques because data fragments consist of a single attribute or multiple attributes. It does not involve data masking or encryption. Hence, the computation is easy. There is another type of encryption in which we do not encrypt and decrypt every time to perform computation. It is called homomorphic encryption. In this case, all data modification is done on encrypted data, and actual data is not changed, however, the final result is preserved [122].

*(3) Steganography*. Steganography is the practice of concealing a message within another message or a physical object. In computing contexts, video, audio, image, message, or computer file is concealed within another image, message, or file. The steganography flow diagram is depicted in Figure 8. There are two main types of steganography, namely (1) linguistic steganography and (2) technical steganography. These techniques are given as follows:

(1) *Linguistic Steganography*
This technique is further divided into two subtechniques, which are given below.
  - *Semagrams*
  - It uses images and symbols alone to cover the data. There are two types of Semagrams [123]. The first is a visual Semagram. In this type, we can visualize the massage. The second type is a text Semagram. In this type, we change the font, color, or symbols of the text message.
  - *Open code*
  - In this case, we hide the real message from the intruder by installing the original massage in an authorized carrier [124]. Open code technique is further divided into two types: one is jargon code, and the second is covered ciphers.
(2) *Technical Steganography*
Technical steganography uses different cover media to hide secret data [125]. There are different types of cover media, such as text, image, audio, and video. Different types of methods are applied on the covers to hide or embed the secret data into the covers.
  (i) Covers
  Cover data is like a vehicle for sending data from one place to another place. Secret messages in cover data exist in two forms: one is streaming, and the second is block [126]. Different types of covers exist, such as text, image, audio, and video. Four different types of steganographic methods are applied on the cover given as blow.
    - *Text steganography*
    - In this type, we change some textual characteristics of text, such as the font, color, or symbols of the text message [127]. Three coding techniques are used to change these textual features, which are as follows: (1) line-shift coding, (2) word-shift coding, and (3) feature coding.
    - *Image steganography*
    - It is the most popular type of steganography. Image steganography refers to the process of hiding sensitive data inside an image file [128]. The transformed image is expected to look very similar to the original image because the visible features of the stego image remain the same. The image steganography is divided into three parts, namely (1) least significant bits coding, (2) masking and filtering, and (3) transformations.
    - *Audio steganography*
    - Audio steganography is a technique that is used to transmit secret data by modifying a digitalized audio signal in an imperceptible manner [129]. Following types of audio steganography are given: (1) least significant bits coding, (2) phase coding, (3) spread spectrum, and (4) echo hiding.
    - *Video steganography*
    - In video steganography, both image and audio steganography are used [130]. A video consists of many frames. Hence, video steganography hides a large amount of data in carrier images. In this type of steganography, we select the specific frame in which we want to hide the sensitive data.
  (ii) Methods
  Two types of methods are used in steganography: (1) spatial domain and (2) frequency domain.
    - *Frequency Domain*
    - A frequency-domain steganography technique is used for hiding a large amount of data with no loss of secret message, good invisibility, and high security [131]. In the frequency domain, we change the magnitude of all of the DCT coefficients of the cover image. There are two types of frequency domain: (1) discrete cosine transformation and (2) discrete wavelet transformation.
    - *Spatial Domain*
    - The spatial domain is based on the physical location of pixels in an image [132]. A spatial domain technique gives the idea of pixel regulation, which minimizes the progressions of a stego image created from the spread image. Some methods of the spatial domain are given as follows: (1) least significant bit, (2) pixel value differencing, (3) pixel indicator, (4) gray level modification, and (5) quantized indexed modulation.

The summary of the steganographic techniques is given in Table 9.

#### 4.1.2. Cryptographic Techniques

Cryptography is the most important and most widely used technique for security purposes. In cryptography, the plain text is converted into ciphertext using a key and some encryption algorithms. Cryptographic techniques are the most secure techniques among all the other security techniques. Hence, these cryptography techniques are widely used in data storage security over the cloud. The present day's cryptography techniques are more realistic. We can achieve different objectives by applying these cryptographic techniques, for example, data confidentiality and data integrity. Because of an increase in the number of data breaches in the last few years, some cloud service provider companies are shifting toward cryptographic techniques to achieve more security. The most commonly used cryptographic technique is AES [133]. Key management is an important issue in cryptographic techniques because if the key is hacked by an intruder, then all the data will be hacked or stolen by this intruder. Hence, key protection or key management is a very important issue. Therefore, it is mostly the responsibility of CSP to manage the key and also provide the protection of key. Cryptographic techniques also protect the user from an untrusted CSP because sometimes the CSP outsources sensitive data without taking the permission of users, and it is an illegal activity. Hence, to avoid these things and protect our sensitive data from untrusted CSPs, we use cryptographic techniques, and it is the best option for users. However, there are some difficulties the user has to face while using cryptographic techniques, i.e., if a user wants to update a small amount of data, the user needs to decrypt the data and then perform this minor update. Hence, this work is very costly. Over time, implementing cryptographic techniques gives us a higher level of security, however, we compromise on performance or speed. It all depends on the user, the standard, the performance, or the high level of security the user wants to achieve. In this paper, we are focusing on the four main functionalities that are required or needed on cloud computing when using cryptographic techniques.  Figure 9 shows the flow diagram of encryption.

Some of the main functionalities of cryptographic functions are given below.

- *Search on encrypted data*
- If a user wants to retrieve their data stored in a cloud database, they generate a query and run the query on a local proxy server and search for the data they want. Searching for encrypted data is a very important part of cryptography because every user who stores their sensitive data in a cloud database wants to retrieve it, and it is done by searching their sensitive data through queries. Therefore, the procedure of retrieving their data is very difficult.
- *Storage control*
- Sometimes the user wants to store data in a desired location or trusted database. Hence, the user must have full control over the storage of data.
- *Access control*
- It is a very important control and is referred to as data access restriction. Sometimes, the user does not want to share a private file publicly. Hence, access control is an important functionality.
- *Computation on data*
- Data computation is the main functionality of cloud computing. Sometimes, the user wants to perform some computation on data that are stored on a cloud database. For example, if a user wants to perform computation on encrypted data that is stored on cloud databases, then there are two ways. One is that the user, firstly, decrypts the entire data, performs computation on the data, and finally, the user encrypts the entire data and stores on the cloud database. This process is very expensive in terms of computation.

Some of the cryptographic techniques are as follows:

*(1) Homomorphic Encryption*. Homomorphic encryption is a form of encryption that permits users to perform computations on encrypted data without decrypting it. These resulting computations are left in an encrypted form, which, when decrypted, result in an identical output to that produced had the operations been performed on the unencrypted data. There are some types of homomorphic encryption that are described below.

- *Partial Homomorphic Encryption*
- In partial homomorphic encryption, only one arithmetic function addition or multiplication is performed at one time. If the resultant ciphertext is the addition of the plain text, then it is called an additive homomorphic scheme, and if the resultant ciphertext is the multiplication of the plaintext, then it is called the multiplicative homomorphic scheme. Two multiplicative homomorphic schemes are given as in [134, 135]. There is one additive homomorphic scheme that is called Paillier [136].
- *Somewhat Homomorphic Encryption*
- This technique allows the user to perform the multiplication and subtraction mathematical operations. However, this scheme allows a limited number of arithmetic operations, because if it allows a large number of arithmetic operations, then it produces noise. This noise changes the structure of the original data. Hence, limited numerical math operations are allowed. There is a somewhat homomorphic encryption scheme that is presented by the authors of the papers [137, 138]. In this scheme, the time of encryption and decryption is increased when multiplication operations are increased. To avoid this increase in time, we allow only a limited number of mathematical operations.
- *Fully Homomorphic Encryption*
- This technique allows a large number of arithmetic operations, namely multiplication and subtraction. Multiplication and addition in this technique are performed in the form of XOR and AND gates [139]. Completely homomorphic encryption techniques require a higher computation time to encrypt and decrypt data. Therefore, this technique is not applicable in real-life applications for implementation. This technique uses a bootstrapping algorithm when a large number of multiplication operations is performed on data and also for the decryption of the data it is used. Homomorphic encryption, on the other hand, represents the trade-off between operations and speed performance. Only a limited number of arithmetic operations are allowed if someone wants low computation, and a large number of arithmetic operations are allowed if someone wants high security. It depends on the needs of the user.

*(2) Searchable Encryption*. A searchable encryption technique is proposed by the author of the paper [140]. In this technique, before storing data on a cloud database, encryption is performed, and after that, it is stored on the cloud. The advantage of this technique is that when we search for some data over the cloud database, this technique provides a secure search over the cloud database.

- *Searchable Asymmetric Encryption*
- Over the past two decades, we have focused on searchable encryption. Much of the work is related to the multiwriter and single-reader cases. Searchable encryption is also called public keyword search encryption along with keyword search (PEKS) [141].
- *Searchable Symmetric Encryption*
- Symmetric-key algorithms use the same key for massage encryption and ciphertext decryption. The keys can be the same, or there can be a simple transformation to go between the two keys. Verifiable searchable symmetric encryption, as a key cloud security technique, allows users to retrieve encrypted data from the cloud with keywords and verify the accuracy of the returned results. Another scheme is proposed for keyword search over dynamic encrypted cloud data with a symmetric-key-based verification scheme [142].

*(3) Encryption*. In cryptography, encryption is the process of encoding information. This process converts the original representation of the information, known as plaintext, into an alternative form known as ciphertext. Ideally, only authorized parties can decipher a ciphertext back to plaintext and access the original information.

- *Symmetric Key Encryption*
- Only one key is used in symmetric encryption to encrypt and decrypt the message. Two parties that communicate through symmetric encryption should exchange the key so that it can be used in the decryption process. This method of encryption differs from asymmetric encryption, where a pair of keys is used to encrypt and decrypt messages. A secure transmission method of network communication data based on symmetric key encryption algorithm is proposed in [143].
- *Public Key Encryption*
- The public-key encryption scheme is proposed by the author of the paper [144]. In this scheme, a public key pair is created by the receiver. This public key pair consists of two keys. One is called a public key, which is known publicly to everyone, and the second is the private key, which is kept a secret. Hence, in this scheme, the sender performs encryption on the data using the public key of the receiver and then sends this encrypted data to the receiver. After receiving this encrypted data, the receiver can decrypt this data using the private key. Hence, in this way, we can perform secure communication between two parties.
- *Identity-Based Encryption*
- Identity-based encryption is proposed by the author of the paper [145]. In this technique, a set of users is registered on the database and a unique identity is assigned to all the registered users by an admin that controls this scheme. The identity of the users can be represented by their name or their e-mail address. Just like in a public-key encryption, there is a public key pair that consists of one public key, which is the identity of the user, and one private key, which is a secret key. Just like in public-key encryption, the receiver cannot generate their public key in identity-based encryption. The identity cannot be generated by the user. There is a central authority that generates and manage the user's identity. The identity-based encryption is improved by the author [146]. The main advantage of identity-based encryption is that anyone can generate the public key of a given identity with the help of the central main authority.
- *Attribute-Based Encryption*
- The authors of the papers [147, 148] propose a technique called attribute-based encryption. Similar to identity-based encryption, attribute-based encryption also depends on the central main authority. The central main authority generates the private key and distributes it to all the registered users. It can be encrypting the messages, however, if it does not have this designation, then it cannot be generating the messages. Attribute-based encryption is used when the number of registered users is very large. Then, the attribute-based encryption is useful. The attribute-based encryption consists of two schemes, which are key policy and ciphertext policy.
- *Functional Encryption*
- A functional encryption technique [149, 150] consists of identity-based encryption, attribute-based encryption, and public-key encryption. All the functionalities of these three techniques combinedly make function encryption. In this technique, all the private keys are generated by the central main authority, which is associated with a specific function. Functional encryption is a very powerful encryption technique that holds all the functionalities of three encryption techniques. A functional encryption technique is used in many applications.

*(4) Signcryption*. Cryptography is publicly open-source, and it functions simultaneously as a digital signature and cipher. Cryptography and digital signatures are two basic encryption tools that can ensure confidentiality, integrity, and immutability. In [151], a new scheme called signature, encryption and encryption is proposed, based on effectively verifiable credentials. The system not only performs encryption and encryption but also provides an encryption or signature form only when needed [152]. The paper proposes lightweight certificate-based encryption using a proxy cipher scheme (CSS) for smart devices connected to an IoT network to reduce computing and communications costs. To ensure the security and efficiency of the proposed CBSS project, we used a cipher system encoded with 80 bit subparameters. Reference [153] proposes an input control scheme for the IoT environment using a cryptographic scheme corresponding to the efficiency and robustness of the UK security system. The proposed scheme shows that besides security services, such as protection against attacks, confidentiality, integrity, nonblocking, nondisclosure, and confidentiality, accounting and communication costs are low compared to the current scheme. Document [154] gives the informal and formal security proof of the proposed scheme. Automated Validation of Internet Security Protocols and Applications (AVISPA) tool is used for formal security analysis, which confirms that the proposed CB-PS scheme can potentially be implemented for resource-constrained low-computing electronic devices in E-prescription systems. The proposed scheme [155] introduced a new concept that does not require a reliable channel. The main production center sends a part of the private key to the public consumers. The summary of the cryptographic schemes is given in Table 10.

All data storage protection on cloud computing is discussed in session 3. There are a lot of data protection techniques, however, all these techniques are only divided into three main categories, namely (i) data splitting, (ii) data anonymization, and (iii) cryptography. From different points views, we discuss all these techniques, e.g., overhead on the local proxy, computation cost, search on encrypted data, data accuracy all these techniques retained, and data protection level all these techniques have, and all the masked data techniques have the functionalities. These are some different views, and by considering them, we can analyze all the data protection techniques. Cryptography provides high-level security but limited cloud functionalities and a high cost of performing computation on cloud data. Data splitting provide low computation cost but a low level of security. Data anonymization is of two types: one is perturbative masking, and the second is nonperturbative masking. Hence, in perturbative masking, data is altered with dummy data. Hence, security is high, however, we cannot perform some functionalities.

### 4.2. RQ2: What are the Demographic Characteristics of the Relevant Studies?

We answer this question by considering the four following aspects: (i) publication trend, (ii) publication venues (proceeding and journals), (iii) number of citations, and (iv) author information.

#### 4.2.1. Publication Trend

From 2010 to 2021, we found 52 papers that were of top ranked journals and conferences. From 2010 to 2017, there is linear work in cloud computing, however, after 2017, a lot of work is done in cloud computing data security. From 2018 to 2021, 37 papers are published. After 2018, the trend about data security in cloud computing increased very vastly. Most of the work is done in 2021. High-ranked studies are published in 2021.  Figure 10 shows all trends of all the publications from 2010. Most of the articles are published in journals venue, and the highest number of papers have been published in IEEE Access journal. 6 papers were published in this journal.

#### 4.2.2. Publication Venues

There are different types of publication venues, and some of them are book articles, conference proceedings, journals, workshop proceedings, and symposium proceedings. Hence, in our SLR, the number of publications in a different venue is given in Figure 11. We have a total of 52 papers after applying the inclusion and exclusion criteria in Section 2.

Out of 52 papers, 0 papers are published in book chapters. 1 paper is published in workshop proceedings. 0 papers are published in symposium proceedings. 43 papers are published in journals. 8 papers are published in conference proceedings. There are some most active journals in cloud data security, which are enlisted in Table 11.

The most active journal is the IEEE Access. In this journal, 6 papers are published. Journal of Cryptology is the second most active journal in the field of data storage, security, and privacy in cloud computing. In this journal, 3 papers are published. In the third journal, i.e., in the Journal of Information Fusion, 3 papers are published. The fourth journal is the Information Science. In this journal, 2 papers are published. The fifth journal is IEEE Transactions on Knowledge and Data Engineering, and in this journal, 2 papers are published. Most active conferences are given in Table 12.

#### 4.2.3. Number of Citations

The number of citations of a paper also tells the quality of the paper. The more the number of citations, the higher the quality, and the fewer the number of citations of the paper, the lower the paper quality.  Table 13 shows the most influential authors, and Figure 12 shows the number of citations of all the papers that we have used in this SLR. Few papers have citations of more than 100. Hence, it shows that papers have a very high quality, and hence, the citation of those papers is very high. These papers are [105, 118, 124, 139].

#### 4.2.4. Author Information

Some authors are most active in their publication. To identify these authors, we enlist the names of the top 10 authors that are more active in the field of data protection and privacy in cloud computing. Hence, we enlist the names of the top 10 authors and also their numbers of publications in Table 13.

### 4.3. RQ3: Which Data Protection Technique Provides More Data Protection among all the Techniques?

We answer this question by considering the following four aspects: (i) publication trend, (ii) publication venues (proceeding and journals), (iii) number of citations, and (iv) author information.

#### 4.3.1. Comparison of Data Protection Techniques

In this section, we compare all the data protection techniques that are discussed in this SLR, and finally, we review which technique is better and provides more protection among all these data protection techniques. We compare these techniques based on different functionalities, which are given as (i) local proxy overhead, (ii) data accuracy retain, (iii) level of data protection, (iv) transparency, and (v) operation supported, and finally, we discuss RQ2.  Table 14 depicts a comparison of all the data protection techniques and provides a brief comparison of all the data protection techniques discussed in this SLR. Now, we discuss all these five functionalities one by one in more detail.

(a) *Local Proxy Overhead*
  1. *Encryption*
  2. The overhead on the local proxy for encryption is very high because the data is encrypted. If the user wants to update the data, firstly, the user decrypts the data and then updates the data. After that, the user encrypts the data again. Hence, this operation requires a lot of time, and all this work is performed by the local proxy. It is the reason the overhead on the local proxy for encryption is very high for encryption.
  3. *Data Splitting*
  4. The overhead on a local proxy for data splitting is very low. The local proxy overhead remains constant while splitting data into fragments.
  5. *Anonymization*
  6. The overhead on a local proxy for anonymization is average because most of the anonymization methods require quasilinear computation in the number of records to generate the anonymized data set. Whenever the anonymized data is generated and stored in the cloud database, then there is no overhead on the local proxy.
  7. *Homomorphic Encryption*
  8. The overhead on local proxies for homomorphic encryption is very high because homomorphic encryption involves a large number of mathematical operations. Therefore, there is a lot of overhead on local proxies for homomorphic encryption.
  9. *Steganography*
  10. The overhead on the local proxy for steganography is not too much as the data is concealed inside the cover for secure communication. However, based on the complexity of the operation in the transformed domain technique, the local proxy overhead is more than the spatial domain technique.
  11. *Signcryption*
  12. The overhead on the local proxy for signcryption is high compared to the simple encryption because in signcryption, hashing and encryption are performed in a single logical step. Because of an extra operation in signcryption, the overhead on the local proxy is higher than the simple encryption.
(b) *Data Accuracy Retain*
  1. *Encryption*
  2. The data accuracy level for encryption is very high because data is encrypted by applying some algorithms. The sensitive data is encrypted by the sender, and this data is decrypted by the receiver using a key. This data cannot be read by anyone who does not have the secret key. Therefore, data accuracy is very high for encryption.
  3. *Data Splitting*
  4. The data accuracy level for data splitting is average because data-splitting data is present in the form of fragments. Therefore, CSP can easily access the fragments of data. Both encryption and data splitting are irreversible methods. Hence, we can retrieve the original data easily.
  5. *Anonymization*
  6. The data accuracy level for data anonymization is very low because anonymization is not irreversible. In anonymization, data is replaced with dummy data, and it cannot be retrieved back. Therefore, anonymization has a very low level of data accuracy.
  7. *Homomorphic Encryption*
  8. The data accuracy level for homomorphic encryption is very high because data is encrypted by applying some algorithms.
  9. *Steganography*
  10. The data accuracy level for steganography is very low as compared to the other cryptographic techniques because data is embedded inside the cover of another medium. Any change in the cover during transmission results in the change of the concealed data. Therefore, it is hard to ensure a high accuracy level in steganography. The stego image contains the secrete data that is transmitted over the communication channel. Data concealed by the sender is extracted from the cover by the receiver. Therefore, the concealment of data results in accurate data transmission.
  11. *Signcryption*
  12. The data accuracy level for signcryption is also very high, because in signcryption, confidentiality and authentication are achieved. Therefore, we can also verify the identity of the sender.
(c) Level *of Data Protection*
  1. *Encryption*
  2. The level of data protection is very high for encryption techniques, because in encryption, data is changed into ciphertext, which cannot be understood. Therefore, we can say that the identification of data is impossible without decryption using a secret key because encryption is a one-way function that is easy to execute in one direction, however, it is impossible to execute in the opposite direction.
  3. *Data Splitting*
  4. The level of data protection for data splitting is less high as compared to cryptographic techniques because data is split into different fragments, and these fragments contain original forms of data. Hence, if an intruder hacks or steal these fragments, then the untired data can be easily read. Hence, the data protection level is not high as compared to encrypted methods.
  5. *Anonymization*
  6. The level of data protection for data anonymization is less high as compared to cryptographic techniques, because in anonymization techniques, quasi-identifiers are protected if the quasi-identifiers are not protected strongly. Then, there is a change in the reidentification of person-sensitive data.
  7. *Homomorphic Encryption*
  8. The level of data protection is very high for homomorphic encryption techniques because encryption data is changed into ciphertext, which cannot be understood.
  9. *Steganography*
  10. The data protection level for steganography is medium because data is embedded inside the cover of another medium. The stego image contains the secrete data that is transmitted over the communication channel. Data concealed by the sender is extracted from the cover by the receiver. Therefore, the concealment of data results in secure data transmission.
  11. *Signcryption*
  12. The data protection level for signcryption is also very high, because in signcryption, both confidentiality and authentication are achieved. Therefore, we can also verify the identity of the sender.
(d) *Transparency*
  1. *Encryption*
  2. There is no transparency for the encrypted data, because in encryption, there is a need for key management. Hence, the local proxy needs to keep the records of all the keys and manage all these keys. Therefore, there is no transparency for the encrypted data.
  3. *Data Splitting*
  4. There is no transparency for the data-splitting mechanism, because in the data-splitting mechanism, data is split into different fragments, and the local proxy stores these fragments in different locations. Hence, there is a need to keep the record of the location of all the fragments that are stored on different locations.
  5. *Anonymization*
  6. Anonymization is fully transparent, because in anonymization, there is no need to keep the record of data storage by the local proxy. In anonymization, data is statistically similar to the original data. Hence, CSP also performs computation and some analysis on the anonymized data.
  7. *Homomorphic Encryption*
  8. There is no transparency for the homomorphically encrypted data, because in encryption, there is a need for key management. Hence, the local proxy needs to keep the records of all the keys.
  9. *Steganography*
  10. In steganography, as compared to other data protection techniques, the main aim is to transmit data without letting the attacker know about the data transmission as it is concealed inside the cover of another medium. The data transmission in steganography is fully transparent. No key management is required, and there is no need to keep track of data storage.
  11. *Signcryption*
  12. There is no transparency for the signcrypted data, because in signcryption, there is a need for key management. Hence, the local proxy needs to keep the records of all the keys and also manage all these keys.
(e) *Operation Supported*
  1. *Encryption*
  2. Only the data storage operation is supported on the encrypted data, because if the user wants to update some encrypted data that are stored on a cloud database, firstly, the user needs to decrypt this data, and then the user performs an update on this data. We cannot perform any modification operation on encrypted data.
  3. *Data Splitting*
  4. All the operations cloud be performed on data splitting, because in data splitting, the data is present in their original structure. Hence, we can perform data storage, search, data update, and also data computation.
  5. *Anonymization*
  6. In anonymization, there are two types of data anonymization: one is data masking, and the second is data nonmasking. If data is nonmasked, then we can perform data storage and search on this data. Otherwise, we can only perform data storage.
  7. *Homomorphic Encryption*
  8. Only the data storage operation is supported on the encrypted data, because if the user wants to update some encrypted data that are stored on the cloud database, firstly, the user needs to decrypt this data, and then the user performs some updates on this data.
  9. *Steganography*
  10. A stego image only supports data storage operations because if the user wants to update the data hidden in a stego image, the user, firstly, retrieves that data from the stego image, and the user can perform any modification on this data.
  11. *Signcryption*
  12. Only the data storage operation is supported on the signcrypted data, because if the user wants to update signcrypted data that are stored on the cloud database, firstly, the user needs to unsign this data, and then the user can perform any update on this data.

## 5. Conclusion and Future Work

### 5.1. RQ4: What are the Primary Findings, Research Challenges, and Direction for Future Work in the Field of Data Privacy in Cloud Computing?

#### 5.1.1. Conclusion and Research Challenges

In this SLR, we have presented all the data privacy techniques related to data storage on cloud computing systematically, and we also present a comparison among all the protection techniques concerning the five finalities, which are the (i) local proxy overhead, (ii) data accuracy retains, (iii) level of data protection, (iv) transparency, and (v) operation supported. There are some research gaps we found in all these techniques of data splitting, anonymization, steganography, encryption, homomorphic encryption, and signcryption.

- There is a very strong need to develop some ad hoc protocols for the communication of data splitting fragments that are stored on different CSPs, and also, there is a strong need to develop some protocol for the communication between different CSPs. Noncryptographic techniques are faster on different CSPs but do not provide enough security. Hence, we can improve security by developing some methods for data-splitting techniques.
- Anonymity techniques work very effectively on a small amount of data but not for big data. Hence, there is a search gap in which we can develop some anonymity techniques to achieve more efficient performance. Therefore, some anonymous schemes need to be developed, which provide stronger protection to the quasi-identifier. Current anonymity techniques are very immature.
- One of the limitations of steganography is that one can only use it to defend against a third party who does not know steganography. If the third party knows steganography, it can extract the data in the same way that the recipient extracts it. Therefore, we always use encryption with steganography. Therefore, there is a need to develop such steganography techniques that can protect sensitive data from third parties.
- There is a need to develop some cryptographic techniques that can take less time than the existing cryptographic techniques to perform search and computation operation on encrypted data. Cryptographic techniques provide high security but low computational utility. Therefore, it is a search gap to develop some techniques that provide both high security with more efficiency.
- The complexity of homomorphic encryption and decryption is far greater than that of normal encryption and decryption, and it is not applicable to many applications, such as healthcare and time-sensitive applications. Therefore, there is an urgent need to develop such homomorphic encryption schemes that have low complexity and computation cost.
- Signcryption is used to verify and authenticate users. We can obtain confidentiality and authentication using signcryption, however, the main limitation of signcryption is that the calculation costs of the encryption algorithm used in signcryption are very high. Therefore, there is a need to develop such signcryption schemes that use such encryption algorithms, which have low computation cost.

## Figures and Tables

**Figure 1:** Review procedure.

**Figure 2:** Study selection procedure.

**Figure 3:** Percentage of selected studies.

**Figure 4:** Taxonomy of the data protection techniques.

**Figure 5:** Data workflow on cloud using local proxy.

**Figure 6:** Data anonymization flow diagram.

**Figure 7:** Data-splitting flow diagram.

**Figure 8:** Steganography flow diagram.

**Figure 9:** Encryption flow diagram.

**Figure 10:** Number of publications per year.

**Figure 11:** Publication venues.

**Figure 12:** Number of citations of the papers.

**Table 1:** Databases sources.

Electronic databases	URL
IEEE xplore	http://ieeexplore.ieee.org/
Wiley	http://onlinelbrary.wiley.com/
Springer link	http://link.springer.com
ACM	http://dl.acm.org/
Elsevier	http://elsevier.com/
Hindawi	https://www.hindawi.com/

**Table 2:** Databases search query.

Database name	Search query
IEEE xplore	((“Document Title”: cloud∗) AND (“Document Title”: data AND (privacy OR protect∗ OR secure∗ OR integrity∗)))
Wiley	“Cloud computing” in Title and “data AND (privacy OR protect∗ OR secure∗ OR integrity∗)” in Title
Springer link	((“Document Title”: cloud∗) AND (“Document Title”: data AND (privacy OR protect∗ OR secure∗ OR integrity∗)))
ACM	acmdlTitle:(+“cloud computing” +data privacy protect∗ secure∗ integrity∗)
Elsevier	((Document Title: cloud computing∗) AND (Document Title: data AND (privacy OR protect∗ OR secure∗)))
Hindawi	((“Document Title” cloud) AND (“Document Title” data AND (privacy OR protect OR secure OR integrity)))

**Table 3:** Results from electronic databases.

Identifier	Database	Initial results	After title screening	After abstract screening	After exclusion and inclusion
ED1	IEEE	942	223	38	24
ED2	ACM	337	127	28	00
ED3	Elsevier	78	52	17	11
ED4	Springer	45	31	18	09
ED5	Wiley	53	45	4	02
ED6	Hindawi	44	9	3	01
ED7	Others	17	15	34	05

**Table 4:** Inclusion and exclusion criteria.

Inclusion criteria	Exclusion criteria
(a). Articles proposing data protection techniques in the context of cloud computing.	(a). Articles other than the English language.
(b). Peer-reviewed articles only.	(b). Articles that are not supported the research questions.
(c). Take the latest study if there are several papers with the same objectives.	(c). Articles providing no validation of proposed techniques.
(d). Comparative studies that compare one or more data protection techniques in cloud computing.	(d). Articles that do not clearly define findings and unbiased results.
(e). Journal papers with impact factors only.	(e). Duplicate studies concerning title or content.
(f). Ranked conference papers only.	(f). Editorials, short papers, posters, technical reports, patents, and reviews.

**Table 5:** Quality checking criteria.

QC1	Are the goals and objectives of the paper described?
QC2	Are there any concise and clear limitations and statements?
QC3	Does the research design support state objectives?
QC4	Is the proposed technique providing any validation?

**Table 6:** Identifiers classification.

Identifier	Categorical	Numerical
Name	✓	×
Age	×	✓
Gender	✓	×
Address	✓	×
Zip-code	×	✓
Designation	✓	×
Salary information	×	✓
Diseases	✓	×

**Table 7:** The summary of data anonymization techniques.

Method	References	Operations supported	Usability	Privacy
Swapping	[99–101]	Research and application testing	Applicable for any type of attributes	
Noise addition	[102]	Research and application testing	Used for the numerical data set	Differential privacy
Microaggregation	[103–105]	Research and application testing	Used for categorical attributes and numerical data sets	*k*-Anonymity. *l*-Diversity. *t*-Closeness
Pseudonymization	[106]	Research and application testing	Used for the numerical data set	
Bucketization	[108]	Research and application testing	Used for categorical attributes and numerical data sets	Segmentation
Slicing	[109]	Research and application testing	Used for categorical attributes	Clustering
Sampling	[110]	Research and application testing	Large utility loss	
Generalization	[111]	Research and application testing	Granularity and utility loss	*k*-Anonymity. *l*-Diversity. *t*-Closeness

**Table 8:** The summary of the data-splitting techniques.

Splitting techniques	References	Operations supported	Usability	Privacy
Byte level splitting	[113]	Storage and retrieval	Useful for binary files. Provides week data privacy	Provides a low level of privacy
Privacy level splitting	[114]	Storage and retrieval	Used for sensitive data. Provides strong protection	Fragments stored on the trusted locations. Provides a high level of privacy
Byte level splitting with replication	[115]	Storage and retrieval	Provides fast retrieval	Data duplication provides low levels of privacy.
Byte level splitting with encryption	[116, 117]	Storage and retrieval	Provides very strong protection	Ciphertext provides a very high level of privacy
Vertical splitting	[118–122]	Storage, retrieval, search, computation	Useful for structural data	Provides a low level of privacy

**Table 9:** The summary of the steganographic techniques.

Steganographic techniques	References	Operations supported	Usability	Privacy
Semagrams	[123]	Storage and retrieval	Only uses images and symbols to cover the data	Provides a low level of privacy
Open code	[124]	Storage	Used to hide the message from the intruder	Low level of privacy as compared to cryptographic techniques
Text steganography	[127]	Storage and retrieval	Used to change some textual characteristics of the text	Very low level of privacy
Image steganography	[128]	Storage and retrieval	Used to hide sensitive data inside an image file	Provides a medium level of privacy
Audio steganography	[129]	Storage and retrieval	Modifying a digitalized audio signal	Provides a high level of privacy
Video steganography	[130]	Storage and retrieval	Uses both image and audio steganography	Depends on the video resolution. Higher the resolution, greater the privacy
Frequency Domain	[131]	Only storage	Hiding a large amount of data with no loss of secret message	Provides a high level of privacy as compared to other steganographic techniques
Spatial Domain	[132]	Storage and retrieval	The used physical location of pixels in an image	Depends on the image resolution. Higher the resolution, greater the privacy

**Table 10:** The summary of the cryptographic techniques.

Cryptography techniques	References	Supported operations	Usability	Privacy
Identity-based encryption	[145, 146]	Use for data access control	Required a valid password to access data	Provides a high level of privacy
Symmetric-key encryption	[143]	Encryption and Decryption of data using the same key	No functionality can be performed on encrypted data	Provides a high level of privacy
Public-key encryption	[144]	Use for data access control	Required a valid public key for encryption and private key for decryption	No key exchange is required. Provides a very high level of privacy
Attribute-based encryption	[147, 148]	Data access control based on attributes	Less secure than public-key encryption	Provides lesser privacy than public-key encryption
Functional encryption	[149, 150]	Used for selected plaintext	Required a valid function	Privacy depends on the function
Fully HE	[139]	Allows all the arithmetic operations	Practically not useable	Provides a very high level of privacy
Somewhat HE	[137, 138]	Allows more addition and one multiplication	Useable for limited arithmetic operations	Provides a medium level of privacy
Partially HE	[134–136]	Allows only one arithmetic operation	Useable for limited arithmetic operations	Provides a low level of privacy
Searchable encryption	[140–142]	Allows query search on encrypted data	Useable on encrypted data	Provides a high level of privacy
Signcryption	[151–155]	Used for user authentication	Useable when efficient authentication is required	Provides a high level of privacy

**Table 11:** Top 5 most active journals.

Title	Number of papers
IEEE access	6
Journal of cryptology	3
Information fusion	3
Information science	2
IEEE transactions on knowledge and Data engineering	2

**Table 12:** Top 5 most active conferences.

Title	Number of papers
International conference on privacy in statistical databases	1
International conference on database systems for advanced applications	1
International conference on high performance and smart computing	1
International conference on mechatronic sciences, electric engineering, and computer	1
Conference on computer vision and pattern recognition	1

**Table 13:** Top 10 most influential authors in data protection in cloud computing.

Name	Institution	Number of papers
Insaf Ullah	Department of information Technology, Hazara University, mansehra 21120, Pakistan	4
Rodríguez-Hoyos A	Departamento de electrónica, telecomunicaciones y redes de Información, escuela politécnica Nacional, ladrón de Guevara	2
Yang JJ	Tsinghua National laboratory for information science and Technology, tsinghua University	2
Ahmad Al Badawi	Faculty of engineering, National University of Singapore, Singapore	1
Nicolas Gama	Laboratoire de mathématiques de versailles	1
Xinrui Ge	X. Ge is with the college of computer science and Technology, Qingdao University	1
Hua Deng	College of computer science and electronic engineering, Hunan University	1
Jiguo Li	Fujian provincial key laboratory of network security and cryptology	1
Gil Segev	School of computer science and engineering, Hebrew University of Jerusalem	1
Andreea B	Department of electrical and systems engineering, University of Pennsylvania	1

**Table 14:** Comparison of data protection techniques.

Techniques	Local proxy overhead	Data accuracy retains	Level of data protection		Transparency	Operation supported	Applicable condition
Encryption	Large overhead on proxy because of encryption and decryption	Provides a high level of data accuracy	Provides a very high level of data protection using encryption		Requires management of key	Only storage	Applicable when user wants high-level security and low-level performance
Anonymization	Quasi-attribute splitting overhead	Low-level data accuracy depends on masking methods	The average level of data protection depends on the anonymization methods	Fully transparent for CSP and local proxy		Storage, search on nonmasked data, and computation	Applicable when testing over the statistical original data is required
Splitting	Remains the same in all operations	Provides a high level of accuracy for the user and CSP	Provides no guarantee about the protection of data fragments		Not transparent for local proxy, keeps record of the fragments' location	All the operation cloud be performed	Applicable when user wants high-level computation performance and low-level data security
Homomorphic encryption	Large overhead on proxy because of large numbers of arithmetic operations	Provides a high level of accuracy	Provides a high level of data protection		Requires management of key	Storage and arithmetic operation computation	Applicable when the user wants high-level computation performance and also high-level data security
Signcryption	Large overhead on proxy because of signcryption and unsigncryption	Provides a high level of data accuracy	Provides a very high level of data protection like confidentiality and authentication		Requires management of key	Only storage	Applicable when user wants data confidentiality and authentication with high protection
Steganography	No overhead on the local proxy	Provides very low accuracy as compared to the other cryptographic techniques	Provides a medium level of data protection		Fully transparent for CSP and local proxy	Only storage	Applicable when the user wants a medium level of data protection with low computation

## Data Availability

The data used to support the findings of this study are provided in this article.

## References

[1] Xiao Z., Xiao Y. (2013). Security and privacy in cloud computing. *IEEE Communications Surveys & Tutorials*.

[2] Khan A. A., Laghari A. A., Awan S., Jumani A. K. (2021). Fourth industrial revolution application: network forensics cloud security issues. *Security Issues and Privacy Concerns in Industry 4.0 Applications*.

[3] Grance M. P. T. (2011). *The NIST Definition of Cloud Computing*.

[4] Karthika A., Muthukumaran N. (2021). An ADS-PAYG approach using trust factor Against economic denial of sustainability attacks in cloud storage. *Wireless Personal Communications*.

[5] Alam T. (2020). Cloud computing and its role in the information technology. *IAIC Transactions on Sustainable Digital Innovation (ITSDI)*.

[6] Sanaei Z., Abolfazli S., Gani A., Buyya R. (2014). Heterogeneity in mobile cloud computing: taxonomy and open challenges. *IEEE Communications Surveys & Tutorials*.

[7] Branch R., Tjeerdsma H., Wilson C., Hurley R., Mcconnell S. (2014). Cloud computing and big data: a review of current service models and hardware perspectives. *Journal of Software Engineering and Applications*.

[8] Cisco Visual Networking Index (2016). *Global Mobile Data*.

[9] Singh A., Chatterjee K. (2017). Cloud security issues and challenges: a survey. *Journal of Network and Computer Applications*.

[10] Praveen K. P., Syam K. P., Alphonse P. J. A. (2018). Attribute based encryption in cloud computing: a survey, gap analysis, and future directions. *Journal of Network and Computer Applications*.

[11] Khan M. A. (2016). A survey of security issues for cloud computing. *Journal of Network and Computer Applications*.

[12] Singh S., Jeong Y.-S., Park J. H. (2016). A survey on cloud computing security: issues, threats, and solutions. *Journal of Network and Computer Applications*.

[13] Tang J., Cui Y., Li Q., Ren K., Liu J., Buyya R. (2017). Ensuring security and privacy preservation for cloud data services. *ACM Computing Surveys*.

[14] Shan Z., Ren K., Blanton M., Wang C. (2018). Practical secure computation outsourcing: a survey. *ACM Computing Surveys*.

[15] Ateniese G., Randal C. B, Reza C Provable data possession at untrusted stores.

[16] Juels A., Kaliski B. S. PORs: proofs of retrievability for large files.

[17] Shacham H., Waters B. Compact proofs of retrievability.

[18] Ateniese G., Di Pietro R., V Mancini L., Tsudik G. Scalable and efficient provable data possession.

[19] Erway C. C., Küpçü A., Papamanthou C., Tamassia R. (2015). Dynamic provable data possession. *ACM Transactions on Information and System Security*.

[20] Yan H., Li J., Han J., Zhang Y. (2017). A novel efficient remote data possession checking protocol in cloud storage. *IEEE Transactions on Information Forensics and Security*.

[21] Shen J., Shen J., Chen X., Huang X., Susilo W. (2017). An efficient public auditing protocol with novel dynamic structure for cloud data. *IEEE Transactions on Information Forensics and Security*.

[22] Liu C., Ranjan R., Yang C., Zhang X., Wang L., Chen J. (2015). MuR-DPA: top-down levelled multi-replica merkle hash tree based secure public auditing for dynamic big data storage on cloud. *IEEE Transactions on Computers*.

[23] Wang H. (2015). Identity-based distributed provable data possession in multicloud storage. *IEEE Trans. Serv. Comput., *.

[24] Li J., Yan H., Zhang Y. (2019). Efficient Identity-Based Provable Multi-Copy Data Possession in Multi-Cloud Storage. *IEEE Trans. Cloud Comput*.

[25] Wang H. (2013). Proxy provable data possession in public clouds. *IEEE Trans. Serv. Comput., *.

[26] Li J., Yan H., Zhang Y. (2021). Identity-based privacy preserving remote data integrity checking for cloud storage. *IEEE Systems Journal*.

[27] Wang C., Chow S. S. M., Wang Q., Ren K., Lou W. (2013). Privacy-preserving public auditing for secure cloud storage. *IEEE Transactions on Computers*.

[28] Yu Y., Au M. H., Ateniese G. (2017). Identity-based remote data integrity checking with perfect data privacy preserving for cloud storage. *IEEE Transactions on Information Forensics and Security*.

[29] Li J., Yan H., Zhang Y. (2018). Certificateless public integrity checking of group shared data on cloud storage. *IEEE Trans. Serv. Comput., *.

[30] Shen W., Yang G., Yu J., Zhang H., Kong F., Hao R. (2017). Remote data possession checking with privacy-preserving authenticators for cloud storage. *Future Generation Computer Systems*.

[31] Wang B., Li B., Li H. Knox: privacy-preserving auditing for shared data with large groups in the cloud.

[32] Wang B., Li H., Li M. Privacy-preserving public auditing for shared cloud data supporting group dynamics.

[33] Liu X., Zhang Y., Wang B., Yan J. (2012). Mona: secure multi-owner data sharing for dynamic groups in the cloud. *IEEE Transactions on Parallel and Distributed Systems*.

[34] Chen L., Li J., Zhang Y. (2020). Anonymous certificate-based broadcast encryption with personalized messages. *IEEE Transactions on Broadcasting*.

[35] Wang B., Li B., Li H. (2015). Panda: public auditing for shared data with efficient user revocation in the cloud. *IEEE Trans. Serv. Comput., *.

[36] Yang G., Yu J., Shen W., Su Q., Fu Z., Hao R. (2016). Enabling public auditing for shared data in cloud storage supporting identity privacy and traceability. *Journal of Systems and Software*.

[37] Wu G., Mu Y., Susilo W., Guo F. Privacy-preserving cloud auditing with multiple uploaders.

[38] Nayak S. K., Tripathy S. (2018). SEPDP: secure and efficient privacy preserving provable data possession in cloud storage. *IEEE Trans. Serv. Comput., *.

[39] Yu J., Hao R. (2019). Comments on” SEPDP: secure and efficient privacy preserving provable data possession in cloud storage. *IEEE Trans. Serv. Comput., *.

[40] Mara G. C., Rathod U., Shreyas R. R. G. (2020). CRUPA: collusion resistant user revocable public auditing of shared data in cloud. *Journal of Cloud Computing*.

[41] Lu X., Pan Z., Xian H. (2020). An efficient and secure data sharing scheme for mobile devices in cloud computing. *Journal of Cloud Computing*.

[42] Yu Y., Mu Y., Ni J., Deng J., Huang K. Identity privacy-preserving public auditing with dynamic group for secure mobile cloud storage.

[43] Sankar L., Rajagopalan S. R., Poor H. V. (2013). Utility-privacy tradeoffs in databases: an information-theoretic approach. *IEEE Transactions on Information Forensics and Security*.

[44] Fung B. C. M., Wang K., Fu A. W.-C., Philip S. Y. (2010). *Introduction to Privacy-Preserving Data Publishing: Concepts and Techniques*.

[45] Langari R. K., Sardar S., Amin Mousavi S. A., Radfar R. (2020). Combined fuzzy clustering and firefly algorithm for privacy preserving in social networks. *Expert Systems with Applications*.

[46] Zhao X., Pi D., Chen J. (2020). Novel trajectory privacy-preserving method based on clustering using differential privacy. *Expert Systems with Applications*.

[47] Casas-Roma J. An evaluation of edge modification techniques for privacy-preserving on graphs.

[48] Rahimi M., Bateni M., Mohammadinejad H. (2015). Extended k-anonymity model for privacy preserving on micro data. *International Journal of Computer Network and Information Security*.

[49] Anjum A., Malik SuR., Choo K. K. R. (2018). An efficient privacy mechanism for electronic health records. *Computers & Security*.

[50] Mohammed N., Chen R., Fung B. C. M., Yu P. S. Differentially private data release for data mining.

[51] Sweeney L. (2002). k-ANONYMITY: a model for protecting privacy. *International Journal of Uncertainty, Fuzziness and Knowledge-Based Systems*.

[52] Friedman A., Wolff R., Schuster A. (2008). Providing k-anonymity in data mining. *The VLDB Journal*.

[53] Fung B. C. M., Wang K., Yu P. S. (2007). Anonymizing classification data for privacy preservation. *IEEE Transactions on Knowledge and Data Engineering*.

[54] Kisilevich S., Rokach L., Elovici Y., Shapira B. (2010). Efficient multidimensional suppression for k-anonymity. *IEEE Transactions on Knowledge and Data Engineering*.

[55] Li J., Liu J., Baig M., Wong R. C.-W. (2011). Information based data anonymization for classification utility. *Data & Knowledge Engineering*.

[56] Geetha P., Naikodi C., Setty S. L. N. (2020). Design of big data privacy framework—a balancing act. *Lecture Notes in Electrical Engineering*.

[57] Dwork C. Differential privacy: a survey of results.

[58] Friedman A., Schuster A. Data mining with differential privacy.

[59] Soria-Comas J., Domingo-Ferrer J., Sánchez D., Megías D. (2017). Individual differential privacy: a utility-preserving formulation of differential privacy guarantees. *IEEE Transactions on Information Forensics and Security*.

[60] Sarathy R., Muralidhar K. (2011). Evaluating Laplace noise addition to satisfy differential privacy for numeric data. *Trans. Data Priv., *.

[61] Hua J., Tang A., Fang Y., Shen Z., Zhong S. (2016). Privacy-preserving utility verification of the data published by non-interactive differentially private mechanisms. *IEEE Transactions on Information Forensics and Security*.

[62] Li X., Yang J., Sun Z., Zhang J. (2017). Differential privacy for edge weights in social networks. *Security and Communication Networks*.

[63] Yazdanjue N., Fathian M., Amiri B. (2020). Evolutionary algorithms for k-anonymity in social networks based on clustering approach. *The Computer Journal*.

[64] Hao Y., Cao H., Hu C., Bhattarai K., Misra S. (2014). K-anonymity for social networks containing rich structural and textual information. *Soc. Netw. Anal. Min., *.

[65] Xu D., Wang R., Shi Y. Q. (2016). An improved scheme for data hiding in encrypted H. 264/AVC videos. *Journal of Visual Communication and Image Representation*.

[66] Yang C.-N., Hsu S.-C., Kim C. (2017). Improving stego image quality in image interpolation based data hiding. *Computer Standards & Interfaces*.

[67] Rabie T., Kamel I. (2017). High-capacity steganography: a global-adaptive-region discrete cosine transform approach. *Multimedia Tools and Applications*.

[68] Jung K.-H. (2018). Data hiding scheme improving embedding capacity using mixed PVD and LSB on bit plane. *Journal of Real-Time Image Processing*.

[69] Qiu Y., Qian Z., Yu L. (2015). Adaptive reversible data hiding by extending the generalized integer transformation. *IEEE Signal Processing Letters*.

[70] Chen H., Ni J., Hong W., Chen T.-S. (2017). High-fidelity reversible data hiding using directionally enclosed prediction. *IEEE Signal Processing Letters*.

[71] Qian Z., Zhou H., Zhang X., Zhang W. (2018). Separable reversible data hiding in encrypted JPEG bitstreams. *IEEE Transactions on Dependable and Secure Computing*.

[72] Lin H.-Y., Hung Y.-M. (2020). An improved proxy Re-encryption scheme for IoT-based data outsourcing services in clouds. *Sensors*.

[73] Dutta P., Susilo W., Duong D. H., Roy P. S. (2021). Collusion-resistant identity-based proxy Re-encryption: lattice-based constructions in standard model. *Theoretical Computer Science*.

[74] Wang D., Sun W., Yu S., Li L., Liu W. (2016). A novel background-weighted histogram scheme based on foreground saliency for mean-shift tracking. *Multimedia Tools and Applications*.

[75] Li M., Li Y. (2017). Histogram shifting in encrypted images with public key cryptosystem for reversible data hiding. *Signal Processing*.

[76] Wang J., Ni J., Zhang X., Shi Y.-Q. (2016). Rate and distortion optimization for reversible data hiding using multiple histogram shifting. *IEEE Transactions on Cybernetics*.

[77] Ni Z., Shi Y.-Q., Ansari N., Su W. (2006). Reversible data hiding. *IEEE Transactions on Circuits and Systems for Video Technology*.

[78] Kumar A., Kumar A. (2016). A cell-array-based multibiometric cryptosystem. *IEEE Access*.

[79] Lee Y., Kim Y.-S., No J.-S. (2017). Ciphertext-only attack on linear feedback shift register-based Esmaeili-Gulliver cryptosystem. *IEEE Communications Letters*.

[80] Belazi A., Khan M., El-Latif A. A. A., Belghith S. (2017). Efficient cryptosystem approaches: S-boxes and permutation–substitution-based encryption. *Nonlinear Dynamics*.

[81] Zhang L., Hu Y., Wu Q. Short signature from the bilinear pairing.

[82] Hussain S., Ullah S. S., Ali I. (2022). An efficient content source verification scheme for multi-receiver in NDN-based Internet of Things. *Cluster Computing*.

[83] Sharma N., Sharma B. K. (2018). Identity-based signature scheme using random oracle model. *Journal of Computer and Mathematical Sciences*.

[84] Yuan E., Wang L., Cheng S., Ao N., Guo Q. (2020). A key management scheme based on pairing-free identity based digital signature algorithm for heterogeneous wireless sensor networks. *Sensors*.

[85] Liu J. K., Baek J., Zhou J., Yang Y., Wong J. W. (2010). Efficient online/offline identity-based signature for wireless sensor network. *International Journal of Information Security*.

[86] Sharma G., Bala S., Verma A. K. (2017). PF-IBS: pairing-free identity based digital signature algorithm for wireless sensor networks. *Wireless Personal Communications*.

[87] Chaudhari P., Das M. L. (2021). PAC: privacy preserving proxy re-encryption for access control in public cloud. *Information Security Journal: A Global Perspective*.

[88] Li K., Zhang W., Yang C., Yu N. (2015). Security analysis on one-to-many order preserving encryption-based cloud data search. *IEEE Transactions on Information Forensics and Security*.

[89] Bansal V., Garg S. (2022). *A Cancelable Biometric Identification Scheme Based on Bloom Filter and Format-Preserving Encryption*.

[90] Watro R., Kong D., Cuti S., Gardiner C., Lynn C., Kruus P. TinyPK: securing sensor networks with public key technology.

[91] Rivest R. L., Shamir R. L., Adleman L., Adleman A. (1978). “A method for obtaining digital signatures and public-key cryptosystems. *Communications of the ACM*.

[92] Diffie W., Hellman M. (1976). New directions in cryptography. *IEEE Transactions on Information Theory*.

[93] Wong K. H. M., Zheng Y., Cao J., Wang S. (2006). A dynamic user authentication scheme for wireless sensor networks. *IEEE International Conference on Sensor Networks, Ubiquitous, and Trustworthy Computing (SUTC’06)*.

[94] Hassan J., Shehzad D., Ullah I. (2021). A lightweight proxy Re-encryption approach with certificate-based and incremental cryptography for fog-enabled E-healthcare. *Security and Communication Networks*.

[95] Keele S. (2007). *Guidelines for Performing Systematic Literature Reviews in Software Engineering*.

[96] Alam K. A., Ahmad R., Akhunzada A., Nasir M. H. N. M., Khan S. U. (2015). Impact analysis and change propagation in service-oriented enterprises: a systematic review. *Information Systems*.

[97] Domingo-Ferrer J., Ricci S., Domingo-Enrich C. (2018). Outsourcing scalar products and matrix products on privacy-protected unencrypted data stored in untrusted clouds. *Information Sciences*.

[98] Kaaniche N., Laurent M. (2017). Data security and privacy preservation in cloud storage environments based on cryptographic mechanisms. *Computer Communications*.

[99] Rodriguez-Garcia M., Batet M., Sánchez D. (2019). Utility-preserving privacy protection of nominal data sets via semantic rank swapping. *Information Fusion*.

[100] Rang W., Yang D., Cheng D. (2021). Dependency-Aware tensor scheduler for industrial AI applications: dymem-an aggressive data-swapping policy for training nonlinear deep neural networks. *IEEE Industrial Electronics Magazine*.

[101] Muralidhar K., Sarathy R., Domingo-Ferrer J. (2014). Reverse mapping to preserve the marginal distributions of attributes in masked microdata. *Privacy in Statistical Databases*.

[102] Rodriguez-Garcia M., Batet M., Sánchez D. (Apr. 2017). A semantic framework for noise addition with nominal data. *Knowledge-Based Systems*.

[103] Rodríguez-Hoyos A., Estrada-Jiménez J., Rebollo-Monedero D., Parra-Arnau J., Forné J. (2018). Does $ k $-Anonymous microaggregation affect machine-learned macrotrends?. *IEEE Access*.

[104] Monedero D. R., Mezher A. M., Colomé X. C., Forné J., Soriano M. (2019). Efficient k-anonymous microaggregation of multivariate numerical data via principal component analysis. *Information Sciences*.

[105] Soria-Comas J., Domingo-Ferrer J., Sanchez D., Martinez S. T-closeness through microaggregation: strict privacy with enhanced utility preservation.

[106] Bouchelaghem S., Omar M. (2020). Secure and efficient pseudonymization for privacy-preserving vehicular communications in smart cities. *Computers & Electrical Engineering*.

[107] Domingo-Ferrer D., Sánchez J., Soria-Comas J. (2016). Database anonymization: privacy models, data utility, and microaggregation-based inter-model connections. *Synth. Lect. Inf. Secur. Privacy, Trust*.

[108] Vasanth S. (2018). Range based queries over order preserving encrypted data. *International Journal of Pure and Applied Mathematics*.

[109] Chung Y., Kraska T., Polyzotis N., Tae K. H., Whang S. E. (2020). Automated data slicing for model validation: a big data-AI integration approach. *IEEE Transactions on Knowledge and Data Engineering*.

[110] Sun L., Ye X., Zhao J., Lu C., Yang M. Bisample: bidirectional sampling for handling missing data with local differential privacy.

[111] Martínez D., Sánchez D., Sánchez S., Valls A., Batet M. (Oct 2012). Privacy protection of textual attributes through a semantic-based masking method. *Information Fusion*.

[112] Steyerberg E. W. (2018). Validation in prediction research: the waste by data splitting. *Journal of Clinical Epidemiology*.

[113] Zhang X., Sun W., Xu T. Data privacy protection using multiple cloud storages.

[114] Dev T., Sen H., Basak M., Ali M. E. An approach to protect the privacy of cloud data from data mining based attacks.

[115] Ali M., Bilal K., Khan S. U., Veeravalli B., Li K., Zomaya A. Y. (2018). DROPS: division and replication of data in cloud for optimal performance and security. *IEEE Trans. Cloud Comput., *.

[116] Gai K., Qiu M., Zhao H. Security-Aware efficient mass distributed storage approach for cloud systems in big data.

[117] Alqahtani H. S., Sant P. A multi-cloud approach for secure data storage on smart device.

[118] Yang J.-J., Li J.-Q., Niu Y. (2015). A hybrid solution for privacy preserving medical data sharing in the cloud environment. *Future Generation Computer Systems*.

[119] Ganapathy V., Thomas D., Feder T., Garcia-Molina H., Motwani R. Distributing data for secure database services.

[120] Ciriani S., De Capitani Di Vimercati V., Foresti S., Jajodia S., Paraboschi S., Samarati P. (2011). Selective data outsourcing for enforcing privacy. *Journal of Computer Security*.

[121] Sánchez M., Batet D. (2016). C-sanitized: a privacy model for document redaction and sanitization. *J. Assoc. Inf. Sci. Technol., *.

[122] Rafique A., Van Landuyt D., Heydari Beni E., Lagaisse B., Joosen W. (2021). CryptDICE: distributed data protection system for secure cloud data storage and computation. *Information Systems*.

[123] Muñoz A., Carracedo J., Álvarez I. A. Hiding short secret messages based on linguistic steganography and manual annotation.

[124] Yang Z.-L., Guo X.-Q., Chen Z.-M., Huang Y.-F., Zhang Y.-J. (2019). RNN-stega: linguistic steganography based on recurrent neural networks. *IEEE Transactions on Information Forensics and Security*.

[125] Kessler G. C., Hosmer C. (2011). An overview of steganography. *Advances in Computers*.

[126] Shyla M. K., Kumar K. S., Das R. K. (2021). Image steganography using genetic algorithm for cover image selection and embedding. *Soft Computing Letters*.

[127] Satir E., Isik H. (2012). A compression-based text steganography method. *Journal of Systems and Software*.

[128] Lu S.-P., Wang R., Zhong T., Rosin P. L. Large-Capacity image steganography based on invertible neural networks.

[129] Chen L., Wang R., Yan D., Wang J. (2021). Learning to generate steganographic cover for audio steganography using gan. *IEEE Access*.

[130] Karthika P., Vidhya Saraswathi P. (2020). IoT using machine learning security enhancement in video steganography allocation for Raspberry Pi. *Journal of Ambient Intelligence and Humanized Computing*.

[131] Patel R., Lad K., Patel M. (2021). Novel DCT and DST based video steganography algorithms over non-dynamic region in compressed domain: a comparative analysis. *International Journal of Information Technology*.

[132] Lakshmi Sirisha B., Chandra Mohan B. (2021). Review on spatial domain image steganography techniques. *Journal of Discrete Mathematical Sciences and Cryptography*.

[133] Joan D., Vincent R. (2002). *The Design of Rijndael: AES-The Advanced Encryption Standard*.

[134] Alexandru A. B., Gatsis K., Shoukry Y., Seshia S. A., Tabuada P., Pappas G. J. (2021). Cloud-based quadratic optimization with partially homomorphic encryption. *IEEE Transactions on Automatic Control*.

[135] Shoukry Y., Konstantinos G, Amr A Privacy-aware quadratic optimization using partially homomorphic encryption.

[136] Catak F. O., Aydin I., Elezaj O., Yildirim-Yayilgan S. (2020). Practical implementation of privacy preserving clustering methods using a partially homomorphic encryption algorithm. *Electronics*.

[137] Xiong L., Dong D., Xia Z., Chen X. (2018). High-capacity reversible data hiding for encrypted multimedia data with somewhat homomorphic encryption. *IEEE Access*.

[138] Badawi A. A., Veeravalli B., Mun C. F., Aung K. M. M. (2018). High-performance FV somewhat homomorphic encryption on GPUs: an implementation using CUDA. *IACR Transactions on Cryptographic Hardware and Embedded Systems*.

[139] Chillotti I., Gama N., Georgieva M., Izabachène M. (2020). TFHE: fast fully homomorphic encryption over the torus. *Journal of Cryptology*.

[140] Gupta B. B., Li K.-C., Leung V. C. M., Psannis K. E., Yamaguchi S. (2021). Blockchain-assisted Secure fine-grained Searchable Encryption for a Cloud-Based Healthcare Cyber-Physical System. *IEEE/CAA J. Autom. Sin*.

[141] Pan X., Li F. (2021). Public-key authenticated encryption with keyword search achieving both multi-ciphertext and multi-trapdoor indistinguishability. *Journal of Systems Architecture*.

[142] Ge X., Jia Y, Hanlin Z (2019). Towards achieving keyword search over dynamic encrypted cloud data with symmetric-key based verification. *IEEE Transactions on Dependable and Secure Computing*.

[143] Cai W., Yao H. (2021). A secure transmission method of network communication data based on symmetric key encryption algorithm. *Wireless Personal Communications*.

[144] Yu Z., Gao C. Z., Jing Z., Gupta B. B., Cai Q. (2018). A practical public key encryption scheme based on learning parity with noise. *IEEE Access*.

[145] Deng H., Qin Z., Wu Q. (2020). Identity-based encryption transformation for flexible sharing of encrypted data in public cloud. *IEEE Transactions on Information Forensics and Security*.

[146] Zhang X., Tang Y., Wang H., Xu C., Miao Y., Cheng H. (2019). Lattice-based proxy-oriented identity-based encryption with keyword search for cloud storage. *Information Sciences*.

[147] Li J., Zhang Y., Ning J., Huang X., Sen Poh G., Wang D. (2020). Attribute Based Encryption with Privacy protection and Accountability for CloudIoT. *IEEE Trans. Cloud Comput*.

[148] Namasudra S. (2019). An improved attribute‐based encryption technique towards the data security in cloud computing. *Concurrency and Computation: Practice and Experience*.

[149] Komargodski I., Segev G. (2020). From minicrypt to obfustopia via private-key functional encryption. *Journal of Cryptology*.

[150] Brakerski Z., Segev G. (2018). Function-private functional encryption in the private-key setting. *Journal of Cryptology*.

[151] Ullah I., Amin N. U., Khan M. A., Khattak H., Kumari S. (2021). An efficient and provable secure certificate-based combined signature, encryption and signcryption scheme for internet of things (IoT) in mobile health (M-health) system. *Journal of Medical Systems*.

[152] Hussain S., Ullah I., Khattak H. (2020). A lightweight and formally secure certificate based signcryption with proxy re-encryption (CBSRE) for Internet of Things enabled smart grid. *IEEE Access*.

[153] Ullah I., Zahid H., Algarni F., Khan M. A. (2021). An Access Control Scheme Using Heterogeneous Signcryption for IoT Environments. *Computers, Materials and Continua*.

[154] Ullah I., Amin N. U., Almogren A., Khan M. A., Uddin M. I., Hua Q. (2020). A lightweight and secured certificate-based proxy signcryption (CB-PS) scheme for E-prescription systems. *IEEE Access*.

[155] Ullah I., Muhammad A. K, Fazlullah K (2021). An Efficient and Secure Multi-Message and Multi-Receiver Signcryption Scheme for Edge Enabled Internet of Vehicles. *IEEE Internet Things J*.

